# Spatial Prediction of COVID-19 in China Based on Machine Learning Algorithms and Geographically Weighted Regression

**DOI:** 10.1155/2021/7196492

**Published:** 2021-10-13

**Authors:** Qi Shao, Yongming Xu, Hanyi Wu

**Affiliations:** School of Remote Sensing & Geomatics Engineering, Nanjing University of Information Science & Technology, Nanjing 210044, China

## Abstract

COVID-19 has swept through the world since December 2019 and caused a large number of patients and deaths. Spatial prediction on the spread of the epidemic is greatly important for disease control and management. In this study, we predicted the cumulative confirmed cases (*CCCs*) from Jan 17 to Mar 1, 2020, in mainland China at the city level, using machine learning algorithms, geographically weighted regression (GWR), and partial least squares regression (PLSR) based on population flow, geolocation, meteorological, and socioeconomic variables. The validation results showed that machine learning algorithms and GWR achieved good performances. These models could not effectively predict *CCCs* in Wuhan, the first city that reported COVID-19 cases in China, but performed well in other cities. Random Forest (RF) outperformed other methods with a CV‐*R*^2^ of 0.84. In this model, the population flow from Wuhan to other cities (WP) was the most important feature and the other features also made considerable contributions to the prediction accuracy. Compared with RF, GWR showed a slightly worse performance (CV‐*R*^2^ = 0.81) but required fewer spatial independent variables. This study explored the spatial prediction of the epidemic based on multisource spatial independent variables, providing references for the estimation of *CCCs* in the regions lacking accurate and timely.

## 1. Introduction

Since December 2019, a novel coronavirus named COVID-19 was first reported in Wuhan, China, and then swept across China. The number of the confirmed cases has exceeded 80,000 with more than 4,000 reported deaths until May 2020 in China. Moreover, the virus has already spread to the world, which is treated as a Public Health Emergency of International Concern (PHEIC). Until May 2020, the number of the confirmed cases of COVID-19 in the world has exceeded 123 million, and the deaths have exceeded 370,000 according to the statistical data released by Johns Hopkins University (JHU) (https://github.com/CSSEGISandData/COVID-19). Compared with SARS [1] and H1N1 influenza [2], the virus is more transmissible and infectious [3, 4].

Since the outbreak of COVID-19, many studies have been conducted on the prediction and impact factors of COVID-19. (1) Some scholars investigated the influence of meteorological factors on the transmission of COVID-19 [5–9]. They collected meteorological factors such as temperature and humidity, then developed models to evaluate the influence of these factors on the number of cases or deaths. (2) Some studies predicted the severity and tendency of epidemic outbreaks based on meteorological variables, population flow, and socioeconomic factors using multiple linear regression (MLP) and Autoregressive Integrated Moving Average (ARIMA) methods [10–12]. (3) Other studies predicted the spread of COVID-19 based on historical case data using Infectious disease dynamics models [13–17] and machine learning algorithms [18, 19]. Susceptible-Infected-Removed (SIR) and Susceptible-Exposed-Infected-Removed (SEIR) first estimate the main epidemiological parameters of COVID-19, such as the basic reproductive numbers *R*_0_, the per day infection mortality, and recovery rates (more than 90% CI) by simulating the transmission process of the epidemic, and then simulate the epidemic trend and predict the number of confirmed cases. Machine learning algorithms such as Convolutional Neural Network (CNN), Long Short-Term Memory (LSTM), Gated Recurrent Unit (GRU), and Autoregressive Integrated Moving Average (ARIMA) were used to predict the trend of COVID-19 based on the daily numbers of cumulative confirmed cases, new cases, and death cases during the outbreak period of COVID-19.

At present, few researches were carried out on the spatial prediction of COVID-19. Due to the differences in epidemic management systems, response policies, and statistical methods in various regions, there may be no reliable case statistics in some regions. Spatial distribution information of the confirmed cases is of great significance for epidemic control, medical resources allocations, and the deployment of epidemic prevention materials. Our study is aimed at exploring the spatial prediction of COVID-19 in mainland China at the city level by GWR and machine learning algorithms, in order to provide an effective way to predict the numbers of cases in some regions without reliable case statistics based on the case data of other regions.

## 2. Materials

### 2.1. Disease Data

The daily number of the cumulative confirmed cases (*CCCs*) during the period from December 2019 to April 2020 were collected from the National Health Committee of China (http://www.nhc.gov.cn/), including *CCCs* of 361 cities in mainland China.  Figure 1(a) shows the temporal variation of *CCCs* during this period. It should be noted that at the end of January, all the provincial-level administrative regions in mainland China launched the first-level response for major public health emergencies. Due to the timely and effective control strategy, the spread of COVID-19 had been contained. Since the end of February, *CCCs* in mainland China tended to stabilize. Given that the number of cases imported abroad is rising since March, the study period is set from January 17 to March 1, 2020, to reduce the impact of imported cases.  Figure 1(b) shows the spatial distribution of *CCCs* during the study period.

### 2.2. Spatial Dataset

In this study, multisource datasets were employed to derive the independent variables for the spatial prediction of COVID-19. The datasets are as follows:

1. Climate data: previous studies have addressed the influence of meteorological factors on the transmission of COVID-19 [12, 20, 21]. ERA5 (https://climate.copernicus.eu/climate-reanalysis), the latest climate reanalysis dataset produced by the European Centre for Medium-Range Weather Forecasts (ECMWF), was used to derive meteorological factors. It provides gridded hourly atmospheric, land-surface and sea-state parameters at 0.25°spatial resolution, with atmospheric parameters on 37 pressure levels.
2. Traffic data: studies have indicated that COVID-19 mainly spreads from person to person through droplets and contacts [22, 23]. Population flow plays a vital role in the distribution and spread of the epidemic. The traffic data was derived from Baidu Migration Map (http://qianxi.baidu.com/), which is an online map developed by Baidu Inc. It provides inbound and outbound traffic volumes for selected cities and dates in China based on cell phone positioning data, which are proportional to the daily number of people traveling between cities.
3. Socioeconomic data: socioeconomic conditions, including economic, medical, and control measures, also affect the spread of the epidemic [12]. The statistical yearbook was collected from the National Bureau of Statistics of China (NBSC) (http://www.stats.gov.cn/tjsj/ndsj/), which contains resident population and gross domestic prod uct (GDP) at the city level.

## 3. Method

### 3.1. Spatial Independent Variables

Relative humidity (Rh) and air temperature at 2 m height (T2m) were derived from the ERA5 reanalysis dataset. The average Rh and T2m of each city were calculated as meteorological indicators. Four city-level traffic features were derived from Baidu Migration Map, including City Migration index (MoveIn), City Emigration index (MoveOut), intracity travel intensity (Travel), and traffic flow from Wuhan to other cities (WP). The geographic distances from other cities to Wuhan (WD) were also calculated. City-level resident population (People) and GDP were derived from the statistical yearbook.  Table 1 shows the summary of the spatial independent variables.

### 3.2. Models

The relationships between the spread of infectious diseases and various factors are multifaceted and complex. Machine learning algorithms have the advantage of fitting high-dimensional complex relationships, which have been introduced into infectious disease research [24–27]. Random Forest (RF), Gradient Boosting Decision Tree (GBDT), and Support Vector Machine (SVM) are widely used machine learning algorithms, which have proved their effectiveness and applicability in many research fields. In addition, *CCCs* is affected by the surroundings, showing obvious spatial heterogeneity and nonstationary distribution characteristics. Geographically weighted regression (GWR) can reveal the spatial nonstationary effect based on a locally weighted regression model. Therefore, RF, GBDT, and SVM and GWR were introduced for the spatial prediction of COVID-19. In addition, traditional partial least squares regression (PLSR) was also used as a comparison.

#### 3.2.1. Random Forest (RF)

RF [28] is an ensemble-learning algorithm that combines a large set of CART decision trees. To construct trees, Bootstrap samples containing *m* samples are drawn randomly with replacement from the training dataset. During the sampling process, some samples (63.2%) appeared multiple times in the bootstrap samples, and some (36.8%) never appeared, which are referred to as out-of-bag (OOB) data. Then, each of the bootstrap samples is used to fit a regression tree, which is independently grown to its maximum size without any pruning process. The splitting criterion of the regression tree is based on the lowest Gini Index. During the process, RF can provide OOB estimate error for each variable by calculating the difference in the mean square errors between OOB data and the samples. Finally, the outputs of all trees are averaged as the predicted value. RF can reduce the overfitting problem and is not sensitive outliers, showing strong generalization ability in practical application.

#### 3.2.2. Gradient Boosting Decision Tree (GBDT)

GBDT is an integrated machine learning algorithm that develops an ensemble of tree-based models by training multiple decision trees in a sequential manner [29]. The core idea is that each iteration fits a regression tree that learns the residuals left by the previous model and thereby decreases the residual along the gradient direction. Therefore, by constantly adjusting and optimizing the weight of the weak learner to make it a strong learner, the loss function can be minimized and optimized. The results of all regression trees are integrated to get the final prediction. GBDT can handle mixed types of data for both classification and regression tasks and is also robust against outliers.

#### 3.2.3. Support Vector Machine (SVM)

SVM is a machine learning method based on the Vapnik-Chervonenkis (VC) theory of statistical learning theory and the principle of structural risk minimization [27, 30, 31]. By using a cost function to measure the empirical risk, it minimizes the regression error between the predicted and actual values. The main basis of SVM is *ε*-insensitive function [32] and Kernel function, since the *ε*-insensitive loss function can disregard errors within a certain range of the true value, thereby maintaining the sparseness and robustness of the fit. And the Kernel function can transform the data into a higher dimensional space to make it possible to perform the linear separation and improve the generalization ability and finally obtain the non-linear learning model in the original low-dimensional space, thus solving the nonlinear regression problem well. The commonly used radial basis kernel function (RBF) was applied in this study.

#### 3.2.4. Partial Least Squares Regression (PLSR)

PLSR is an effective multivariate statistical method to deal with many and highly collinear predictors [33]. By combining advantages of principal component analysis (PCA) and multiple regression, it is superior to the general linear regression method when analyzing the linear relationships between multiple independent and dependent variables [34]. First, a set of latent factors that explain as much of the covariance as possible between the independent and dependent variable are extracted. Then, a regression model is developed to predict the dependent variable using the latent factors as input variables.

#### 3.2.5. Geographically Weighted Regression (GWR)

According to Tobler's First Law of Geography, everything is spatially related and the closer the distance, the greater the spatial correlation between things [35]. GWR is an expansion of the classical regression that effectively addresses spatial heterogeneity by enabling the coefficients to vary with the spatial locations [36, 37]. GWR formula is as follows:

(1) $$\begin{array}{c} Y_{i}=\beta_{0}\left(u_{i},v_{i}\right)+\overset{p}{\underset{j=1}{\sum }}\beta_{j}\left(u_{i},v_{i}\right)X_{ij}+\in i, \end{array}$$

where *i* is the *i*^th^ city, *Y*_*i*_ is the dependent variable, *β*_0_(*u*_*i*_, *v*_*i*_) is the intercept constant, *p* is the total number of independent variables, *X*_*ij*_ is the *j*^th^ independent variable, *ϵ*_*i*_ is the error term, and *β*_*j*_(*u*_*i*_, *v*_*i*_) represents spatial location function, which can reflect the law of dependent variable changing with geographical location.

GWR is originally developed assuming a Gaussian distribution of the dependent variable, and the weight is determined by Gaussian function as follows:

(2) $$\begin{array}{c} W_{ij}≕\begin{array}{c} \frac{\sqrt{1}}{2\pi }\exp\left(-\frac{1}{2}{\left(\frac{d_{ij}}{h}\right)}^{2}\right),\;d_{ij}<h,\\ 0,\;d_{ij}\geq h, \end{array} \end{array}$$

where *d*_*ij*_ represents the distance between points *i* and *j* and *h* represents the bandwidth and is selected by Corrected Akaike information criterion (AICc), which can avoid overfitting and determine a more reasonable bandwidth [38, 39]:

(3) $$\begin{array}{c} \text{AICc}\left(h\right)=\log\left(\frac{1}{2}{\overset{\wedge }{\in }}^{T}\hat{\in }\right)+\frac{n+\text{tr}\left(L\left(h\right)\right)}{n-2-\text{tr}\left(L\left(h\right)\right)}, \end{array}$$

where *n* is the observed index number, ${\overset{\wedge }{\epsilon }}^{T}\epsilon$ is the error estimation/standard deviation, and tr(∗) is the trace of *L*(*h*), which represents the bandwidth function.

### 3.3. Model Training and Validation

In order to reduce the influence of the wide range of *CCCs* and avoid possible negative values in the predicted results, a logarithmic transformation was applied to *CCCs*:

(4) $$\begin{array}{c} CCCs\text{Log}=\ln\left(CCCs+1\right), \end{array}$$

where *CCCs* is the cumulative confirmed cases at the city level, *CCCs*Log is the logarithmic-transformed *CCCs*. *CCCs* of some cities were zero, *CCCs* plus 1 to avoid the invalid value of ln(0).

*CCCs*Log was used as the dependent variable, and 9 variables (Rh, T2m, MoveIn, MoveOut, Travel, WP, WD, GDP, and People) of each city were used as the independent variables to fit RF, GBDT, SVM, GWR, and PLSR models. The whole dataset contains 361 samples (361 cities in mainland China). 10-fold cross-validation was used to assess the model performances. The whole dataset is randomly divided into 10 subsets (folds), each of which (containing 36 samples) is the test set and the remaining folds (containing 325 samples) are used as the training set. The model developed from the training set is validated based on the test set. This process is repeated 10 times to ensure that each fold is selected as the test set, and all the predicted results of 10 times are compared with actual values. Root mean square error (RMSE), mean absolute error (MAE), and *R*^2^ were calculated as the accuracy indicators. During the modeling, feature selection was also conducted to determine the optimal feature combination.

The predicted values were exponentially transformed to the estimated number of cumulative confirmed cases.

(5) $$\begin{array}{c} CCCsE=\text{INT}\left[\exp^{CCCs\text{Log}}-1\right], \end{array}$$

where *CCCsE* is the estimated cumulative confirmed cases and INT [*x*] represents the maximum integer not exceeding *x*.

SHapley Additive Planations (SHAP) is a game theoretic approach to explain the output of machine learning models. It connects optimal credit allocation with local explanations using the classic Shapley values from game theory and their related extensions [40]. Traditional feature importance only indicates which feature is important but does not show how that feature affects the prediction result. The SHAP value can reflect the influence of the features in each sample and also show the positive and negative effects [41], providing a good way to help understand the impact of independent variables on the model.

## 4. Results and Discussion

### 4.1. Model Performance

The evaluation results of all the models are shown in Table 2. Three machine learning models achieved relatively low CV-RMSE and CV-MAE but also showed extremely low CV‐*R*^2^. Moreover, CV-RMSE of these models were obviously higher than CV-MAE. We carefully analyzed the estimated *CCCs* and found that it can be mostly attributed to Wuhan. Wuhan is the first city that reported COVID-19 cases in China and had an extremely high *CCCs* (49,122). As a contrast, the second and third highest city-level *CCCs* in mainland China were 3,518 and 2,905, respectively. The large difference between *CCCs* of Wuhan and other cities led to serious underestimation of Wuhan and resulted in poor overall accuracy. As for GWR and PLSR, CV‐*R*^2^ were very high (0.98) but CV-RMSE and CV-MAE were also too high. In-depth analysis on the predictions of GWR and PLSR indicated that this was also attributed to Wuhan. GWR generates local regression models at different locations. For Wuhan and its surrounding areas, the developed regression model could not well predict *CCCs* of Wuhan because of the special condition of this city. The seriously overestimated *CCCs* of Wuhan led to the extremely high error. PLSR extracts the principal components of independent variables and then uses Canonical correlation analysis (CCA) and MLP to generate the prediction model. Its predicted results are easily affected by extreme values such as Wuhan and its surrounding cities. In addition, PCA discards nonprincipal components with a small variance which may contain important information and would have a negative impact on subsequent modeling.

Based on the above analysis, Wuhan had great effects on the prediction accuracies of all these models. We removed the predicted *CCCs* of Wuhan from the results and recalculated CV-RMSE, CV-MAE, and CV‐*R*^2^ of all models (Table 3). The performances of all models were obviously improved. CV‐*R*^2^ ranged from 0.37 to 0.84, CV-RMSE ranged from 135.57 to 2,344.51, and CV-MAE ranged from 34.59 to 212.67. Among these models, RF achieved the highest accuracy (CV‐*R*^2^ = 0.84, CV‐MAE = 34.59, and CV‐RMSE = 135.57). GWR had relatively lower accuracy compared with machine learning algorithms. However, GWR used much fewer independent variables based on feature selection, which included WP, WD, MoveIn, MoveOut, and Travel. As a contrast, RF used all the 9 independent variables. PLSR showed the lowest CV‐*R*^2^ and the highest CV-MAE and CV-RMSE, suggesting that it is not suitable for the spatial prediction of the epidemic in our study.

We also validated the performances of these models developed from the dataset of all the other 360 cities (excluding Wuhan). The accuracies were similar to that of Table 3. To save space, we do not give detailed results.

### 4.2. Prediction Error Analysis

Figure 2 gives the predicted results of RF and GWR. Compared with the distribution of actual *CCCs* (Figure 1(b)), the estimated *CCCs* of RF (Figure 2(a)) and GWR (Figure 2(b)) generally showed similar patterns. *CCCs* in mainland China had obvious spatial distribution characteristics, which were very high in the surrounding cities of Wuhan and then decreased with distance to Wuhan. Provincial capital cities exhibited obvious high *CCCs* compared with other cities in the provinces, and Western cities generally had low *CCCs* compared with eastern cities. Figures 2(c) and 2(d) show the scatter plots between actual *CCCs* and estimated *CCCs* of RF and GWR, respectively (excluding Wuhan).

Most of the samples clustered near the 1 : 1 line, suggesting good consistency between the actual and estimated *CCCs*. There were also some overestimated and underestimated samples, marked pink and cyan, respectively, in the plots. Compared with RF, GWR had more outliers in the estimated results. Especially for the cities with high *CCCs*, GWR tended to underestimate *CCCs*.

We noticed that there were some samples with relatively high bias in RF and GWR. To better understand the spatial pattern of prediction error, the distributions of the absolute error of RF and GWR are shown in Figure 3. The spatial characteristics of the prediction error and the possible reasons were discussed as follows.

#### 4.2.1. RF

Package treeinterpreter (https://github.com/andosa/treeinterpreter) can interpret Random Forest predictions and allow decomposing each prediction into bias and feature contribution components that can see which features contributed to the difference and by how much. Based on the outputs from tree interpreter, we found that WP was the most contributing feature. So we focus on analyzing the prediction error from the perspective of WP, as shown in Figure 4.

Some underestimated cities are close to or far from Wuhan with relatively low WP (<0.40). These cities are marked red in Figure 4 and listed in Table 4. Lower WP tends to lead to the underestimation, which can be attributed to the following reasons:

1. Statistical errors in Baidu Migration Map: Baidu Migration data is mainly derived based on cell phone positioning data. However, if people do not use smartphones or any Baidu-related apps or the signal is not good, their migration will be not recorded, resulting in a lower WP value.
2. Multistage spread of the epidemic between cities: though many cities do not have direct large population flows with Wuhan, the epidemic may spread to them through other cities. However, at this stage, we lack the features able to characterize the multi-stage link between cities.

Also, there are some obviously overestimated or underestimated cities with relatively high WP (>0.65). These cities are marked pink and cyan in Figure 4 and listed in Table 5. Most of them belong to or are close to Hubei Province (Wuhan is the capital city of this province). The others are generally other provincial capital cities. It is worth noting that *CCCs* in these cities with similar WP show different *CCCs*, such as Beijing vs. Jiujiang, Zhengzhou vs. Shenzhen vs. Shanghai, and Yichang vs. Xiantao. Some cities with serious epidemics had relatively low WP values, while some cities with mild epidemics had relatively high WP values, which might mislead RF to make wrong predictions. In addition, due to the different management and control capabilities of different cities, the cities with similar independent variable values might have obviously different *CCCs*, which also introduced difficulties for the prediction.

#### 4.2.2. GWR

As shown in Figure 3(b), cities with large prediction errors mainly are the cities with much higher or lower *CCCs* than the surrounding cities. Most of them are the cities in Hubei Province (Xiaogan, Huanggang, Suizhou, Jingzhou, Xiangyang, Ezhou, Huangshi, Yichang, Xianning, Jingmen, Shiyan, Tianmen, Xiantao, Shennongjia, and Enshi); municipalities (Beijing, Shanghai, Chongqing, and Tianjin); provincial capital cities (Haerbin, Guangzhou, Hefei, Zhengzhou, Chengdu, Nanjing, and Changsha); and other cities (Wenzhou, Jining, Shenzhen, Ningbo, Bozhou, Bengbu, Xinyang, Shaoyang, Ganz, and so on). GWR is essentially a combination of local linear regression models, and *CCCs* of each sample is estimated by the surrounding samples. In those outliers' regions, there will be large absolute errors.

### 4.3. Discussion

#### 4.3.1. Feature Importance Analysis

The feature SHAP and importance of the 9 independent variables used in RF are shown in Figure 5. WP is the most important feature. Wuhan is the first city that reported COVID-19 cases in China and the population flow of this city played a vital role in the epidemic spread. MoveOut, MoveIn, and Travel mainly reflect the intensity of population flow between and within cities. These features do not show obvious positive effects on the increase of *CCCs*, which can be attributed to the Chinese government's control policy that restricted residents' travel since January 25, 2020. Resident population and GDP mainly reflect the development level and the intensity of human activities. The epidemic is more serious in those economically developed cities. WD characterizes the geographical distance between each city and Wuhan. However, transportation is much more convenient than before, and remote distance is no longer the main reason for preventing population flow. Weather conditions (Rh and T2m) also show impacts on the epidemic spread, which are not as important as population migration because COVID-19 is mainly spreading through people's contact.

#### 4.3.2. Advantages and Limitations

Previous studies on COVID-19 mostly focused on temporal prediction but little attention was paid to spatial prediction. And previous studies seldom combined machine learning algorithms and spatial data for the spatial prediction of the epidemic. This study explored the potential of machine learning algorithms in the spatial prediction of COVID-19 and compared them with PLSR and GWR. The results show that machine learning algorithms and GWR worked well in the spatial prediction of CCCs at the city level. Machine learning algorithms can achieve the best results, and GWR can obtain good accuracy with fewer independent variables, indicating the applicability of machine learning algorithms and GWR in epidemic prediction. It should be noted that all the models cannot effectively predict *CCCs* in Wuhan, which has obviously negative effects on the overall prediction accuracy. For the other cities, these algorithms performed well. Among all the models, RF achieved the highest accuracy but required more independent variables. With abundant spatial datasets, RF is a good choice for the spatial prediction of *CCCs*. Compared with RF, GWR had a relatively lower accuracy but required fewer variables. If there are no abundant spatial datasets, GWR could be considered for the spatial prediction of *CCCs*.

Reliable spatial distribution information of the confirmed cases is of great significance for epidemic prevention and control. Due to the shortage of COVID-19 testers and medical workers, some regions may not be able to collect accurate and timely information of cases. With the case data of other regions, spatial prediction can provide valuable estimation of the confirmed cases in these regions.

There are also some limitations in this study:

1. Limitation of datasets: due to the lack of datasets at the county level, we conducted studies at the city level. The relatively large spatial scale and small sample size at the city level may have some influence on the modeling, such as overfitting.
2. Not introducing time-dependent variables: the spatial distribution of the epidemic is time-dependent, but we only used nontime series models and did not consider the time-dependent factors.
3. Not using spatial-temporal models: many cities, especially the remote small cities, do not have large and direct people flow with Wuhan. The epidemic may spread to these cities through other cities. Population flow between cities can be represented as a directed graph, and graph Convolutional Neural Networks can automatically learn the characteristics of nodes and the associated information between nodes. With the accurate movement trajectory and location information of people, a directed graph can be generated. Spatiotemporal Graph Neural Networks can combine time-series variables and spatial features to realize the spatiotemporal prediction.
4. Quantification of control measures on the epidemic: since the outbreak of COVID-19, the Chinese government has taken a series of measures to control the epidemic, such as the lockdown of Wuhan, traffic control, closing factories, and stores, allocating epidemic prevention materials, strengthening antiepidemic publicity, and so on. These measures have played a vital role in the epidemic prevention. However, we failed to find an effective way to quantify these measures. If quantitative indicators could be proposed to depict these control measures, the spatial prediction of *CCCs* is expected to be improved.

At last, we shall acknowledge that there are uncertainties during the spread of the epidemic. Quantitative models can predict the cases to a great degree but cannot provide extremely accurate estimations for all cities.

## 5. Conclusion

In this study, the spatial prediction of COVID-19 at the city level in mainland China was conducted using three machine learning algorithms, PLSR, and GWR with multisource spatial variables. The machine learning and GWR models achieved good performance (excluding Wuhan), but the PLSR model achieved a poor performance. RF showed the best accuracy with a CV‐*R*^2^ of 0.84. For the RF model, WP was the most important feature and the other features also made considerable contributions to the prediction accuracy. Compared with RF, GWR showed a relatively lower accuracy with a CV‐*R*^2^ of 0.81, but it had the advantage of requiring fewer independent variables.

All the spatial prediction used for the spatial prediction of the epidemic can be timely obtained from the internet, so the proposed idea and methods in this study can be conveniently applied. This paper provides a template for the spatial prediction of the epidemic in the regions lacking accurate epidemic statistics, which is valuable for the decision-making of anti-COVID-19.

## Figures and Tables

**Figure 1:** (a) The temporal variation of *CCCs* in mainland China from December 1, 2019, to April 30, 2020. The green dotted line represents the start date of study period 2020-01-17, purple represents the end date of study period 2020-03-01, and orange represents the control date of China 2020-01-25. (b) The spatial distribution of city-level *CCCs* in mainland China from January 17 to March 1, 2020.

**Figure 2:** Predicted results of RF and GWR. (a, b) The spatial distributions of the estimated *CCCs* of RF and GWR. (c, d) Scatter plots between actual *CCCs* and estimated *CCCs* of RF and GWR. Pink and cyan marked areas represent obviously overestimated and underestimated samples, respectively.

**Figure 3:** Spatial distribution of the absolute error of RF (a) and GWR (b). Pink and cyan marked areas represent overestimated and underestimated cities, respectively.

**Figure 4:** Spatial distribution of WP in China at the city level. Red marked areas represent the obviously underestimated cities by RF with relatively low WP (<0.40). Pink and cyan marked areas represent the obviously overestimated and underestimated cities by RF with relatively high WP (>0.65).

**Figure 5:** Feature SHAP and importance. (a) SHAP values of every feature in each sample. The plot sorts feature by the sum of SHAP value magnitudes over all samples, which can show the distribution of the impacts each feature has on the model output. The color represents the feature value (red high, blue low). (b) Feature importance.

**Table 1:** Summary of spatial independent variables.

Variables	Description	Data source	Format
Rh^1,∗^	Relative humidity	ERA5	Hourly
T2m^1,^^∗^	Temperature at 2 m height	ERA5	Hourly
MoveIn^∗^	City Migration index	Baidu Migration Map	Daily
MoveOut^∗^	City Emigration index	Baidu Migration Map	Daily
Travel^∗^	Intracity travel intensity	Baidu Migration Map	Daily Daily
WP^2,^^∗^	Traffic flow from Wuhan to other cities	Baidu Migration Map	Daily
WD^3^	Geographic distance from each city to Wuhan	—	Yearly
GDP	GDP per city	NBSC	Yearly
People	Resident population per city	NBSC	Yearly

^1^Calculation of daily average weather variables for each city. ^2^WP is constructed by multiplying MoveOut of Wuhan with percentage that a destination city receives from Wuhan for each Chinese city. For Wuhan, we set the percentage = 100%. ^3^WD is constructed by calculating the geographic distance from each city to Wuhan under UTM ZONE 49N projection. For Wuhan, we set WD = 0. ^∗^Calculation of the average of independent variables for each city from January 17, 2020, to March 1, 2020.

**Table 2:** Evaluation results of machine learning algorithms, PLSR, and GWR.

Model	CV-RMSE	CV-MAE	CV‐*R*^2^
RF	2,503.24	166.05	0.21
GBDT	2,550.63	175.17	0.12
SVM	2,586.37	180.22	0.01
PLSR	2.70∗10^19^	1.42∗10^18^	0.98
GWR	5.82∗10^13^	3.06∗10^12^	0.98

**Table 3:** Evaluation results of machine learning algorithms, PLSR, and GWR without Wuhan.

Model	CV-RMSE	CV-MAE	CV‐*R*^2^
RF	135.57	34.59	0.84
GBDT	178.10	41.37	0.82
SVM	140.20	44.42	0.81
PLSR	2,344.51	212.67	0.37
GWR	194.01	52.98	0.81

**Table 4:** Obviously underestimated cities with relatively low WP (*<*0.40).

City	WP	Observed *CCCs*	Estimated *CCCs*
Xinyu^1^	0.0003	130	7
Bengbu^1^	0.0004	160	10
Huaian^1^	0.0035	66	20
Ningbo^1^	0.0165	157	31
Jining^1^	0.0947	260	34
Bozhou^1^	0.1625	108	41
Taizhou^1^	0.1819	146	53
Fozhou^1^	0.2268	72	34
Shangrao^1^	0.2710	123	45
Hangzhou^1,∗^	0.2889	169	86
Shaoyang^1^	0.3267	102	44
Wenzhou^1^	0.3495	504	98
Jixi^2^	0.0000	46	8
Shuangyashan^2^	0.0000	52	6
Ganz^2^	0.0000	78	2
Suihua^2^	0.0001	47	11
Tangshan^2^	0.0014	58	22
Zhongshan^2,∗^	0.0203	66	27
Zhuhai^2^	0.1561	98	42
Tianjin^2,∗^	0.1661	136	47
Haerbin^2,∗^	0.2112	198	40

^1^Cities close to Wuhan, WD < 700 km. ^2^Cities far from Wuhan, WD > 700 km. ^∗^Municipalities and capital cities.

**Table 5:** Obviously overestimated or underestimated cities with relatively high WP (>0.65).

City	WP	Observed *CCCs*	Estimated *CCCs*
Xianning^1,†^	9.0345	836	1,158
Jingmen^1,†^	6.1535	925	1,213
Xiantao^1,†^	5.4869	575	1,031
Enshi^1,†^	4.0948	252	491
Qianjiang^1,†^	1.9928	198	425
Nanyang^1^	1.2508	156	264
Jiujiang^1^	0.8113	118	212
Zhengzhou^1,∗^	0.7422	157	262
Xiaogan^1,†^	26.2352	3,518	1,736
Huanggang^1,†^	26.0067	2,905	1,621
Jingzhou^1,†^	12.2395	1,579	905
Ezhou^1,†^	6.8330	1,391	1,065
Suizhou^1,†^	5.7935	1,307	1,174
Yichang^1,†^	5.5920	931	734
Shiyan^1,†^	3.8053	672	416
Chongqing^1,∗^	1.8785	576	270
Beijing^2,∗^	0.8908	414	275
Shenzhen^2,∗^	0.7387	417	319
Shanghai^1,∗^	0.7329	337	224
Nanchang^1^	0.7036	230	167
Guangzhou^2,∗^	0.6845	346	281

^1^Cities close to Wuhan, WD < 700 km. ^2^Cities far from Wuhan, WD > 700 km. ^∗^Municipalities and capital cities. ^†^Cities in Hubei province.

## Data Availability

The Data used to find the study can be available from the following links: https://github.com/CSSEGISandData/COVID-19, http://www.nhc.gov.cn/, and http://qianxi.baidu.com/.
